The article "Evaluating Organ Donation Decision in ICU Patients' Families by Analytic Network Process Approach" was published in 2022. Journal: J Healthc Eng.

# Evaluating Organ Donation Decision in ICU Patients' Families by Analytic Network Process Approach

**DOI:** 10.1155/2022/9969604

**Published:** 2022-04-15

**Authors:** Chia-Lun Lo, Hsiao-Yun Chang, Guang-Mao Lee

**Affiliations:** ^1^Department of Health-Business Administration, Fooyin University, Kaohsiung City 83102, Taiwan; ^2^Department of Nursing, Chang Gung University of Science and Technology, Taoyuan City 33303, Taiwan; ^3^Department of Nursing, Kaohsiung Municipal United Hospital, Kaohsiung City 80457, Taiwan

## Abstract

The imbalance between supply and demand for organs has been a global crisis, despite the efforts of transplant coordinators from healthcare institutions to promote donor registration. Because the patient's family has legal rights over the patient's remains, they can easily undermine any efforts spent on organ procurement by simply refusing the patient's consent before death in practice. Most related studies seldom mention the decision-making on organ donation from patients' families. The objectives of this study are to find what are the priorities of those factors acting as the pillars of organ donation by patients' families. This study applied the analytic network process (ANP) to the prioritization factors contributing toward the willingness of families to donate organs of intensive care unit patients. The purposive sampling method used structured questionnaires and ANP questionnaires to enroll 180 patients' families from five intensive care units who met the criteria in the regional teaching hospital of southern Taiwan. Through the ANP analysis, it was found that when family members made organ donation decisions, the weights of the four domains are as follows: psychology—47.6%, externality—20.3%, spirituality—19.7%, and physiology—12.3%. The main decision-making factors that influenced the weighting factors were “attitude” (31.5%), “physician's experience” (0.88%), “religion” (19.3%), and “organ selection” (31.9%). These results could assist organ donation teams to take the best strategies for persuading people to agree with organ donation and formulating an individual organ donation plan.

## 1. Introduction

According to the 2017 data of the Health Resources and Services Administration, an agency of the US Department of Health and Human Services, only 33,612 (28.16%) of the 119,362 individuals awaiting organ transplant have successfully received the transplant. The widening gap between the number of organ donors and recipients is a considerable challenge for governments worldwide. In Taiwan, the Human Organ Transplant Act, which was promulgated in 1987, clearly stipulates that a transplant operation must be performed only after the organ donor has been certified dead by his/her attending physician. Typically, brain death is used as a legal definition of death, and the guidelines for the determination of brain death specify that brain death must be determined when the individual in question is in an intensive care unit (ICU) and is receiving constant perfusion through life support equipment capable of monitoring the individual's hemodynamic parameters. The organs of an individual who is confirmed as brain dead can be donated with the individual's prior consent or with his/her family's consent. Different systems and laws govern organ donation throughout the world, including opt-out (presumed consent) and opt-in presumptive approaches. In fact, in most countries, such approaches are often not rigorously applied because health-care staff members have the family's well-being at heart. Caring for a bereaved family who is going through the unique and distressing experience of a loved one being pronounced brain dead is a responsibility for health-care staff.

The patient's wishes determine the organ donation process. If the patient's wishes are unknown, health-care staff in the given institution deems that decisions should be made by the patient's family. Difficulties can also emerge when the wishes of the patient are inconsistent with those of the patient's family because health-care staff members are obliged to follow the wishes of the patient, potentially creating legal or ethical tensions with the patient's family [1]. In practice, because the patient's family members have legal rights over the patient's remains, they can easily undermine any efforts expended on organ procurement by refusing consent on behalf of the patient before death [2, 3]. Therefore, identifying the factors that affect family consent to organ donation is of utmost importance.

However, the situation is complex, with the family obliged to make decisions about organ donation within a short time despite needing to discuss the matter with other relatives and friends. Extensive communication and explanation tend to characterize this stage of the organ donation process. Identifying which opinion is the most legitimate one among those of relatives is difficult [4, 5]. Family members' subjective opinions on organ donation can also be influenced by their distinct social, cultural, and religious backgrounds. Some studies have noted that families' education level, funerary customs, and openness of communication with medical personnel are factors affecting their decisions about a patient's organ donation [6, 7]. Family members thus play a key role in the decision on whether the patient's organs will be donated because they overrule the patient's wishes in some cases.

Knowledge of the patient's wishes is generally the strongest and most consistent predictor of donation. A family's awareness of its relative's donation wishes is strongly associated with honoring those wishes [8–16]. In addition, studies on organ shortage have generally focused on ICU nursing personnel's attitude toward and knowledge of organ donation, indicating that individuals with extensive organ knowledge and a positive attitude are more inclined to accept organ donation than others [7, 17–19]. Siminoff et al. [18] reported that attitude toward organ donation varied by professional background; a positive attitude toward and consenting to organ donation were positively correlated among individuals from a medical background. Notably, up to 78.3% of the respondents to a survey deemed their immediate family members to be the only ones (apart from themselves) with the right to decide whether their organs might be donated [18]. Nevertheless, a patient's family refusing to comply with the patient's wishes for organ donation despite that patient signing an organ donor card is not an uncommon situation in clinical settings, especially given that the law protects the rights of patients' families over the patients' remains. Therefore, identifying the factors affecting families' decisions regarding organ donation at the critical moment is crucial to the success of organ procurement and could help organ procurement coordinators and medical staff minimize family distress, fulfil the patient's wishes, and increase the rate of organ donation.

The literature does not provide sufficient evidence to determine the opinions of patients' families in deciding on donating organs of their family member. Making a quick decision on whether to donate the organs of a loved one is a difficult, complicated, and multifaceted process. In this study, we assigned weights to the main factors affecting organ donation decisions made by families of ICU patients. Moreover, the relevant literature on psychological factors and cause-and-effect relationships (the qualitative and quantitative perspectives, respectively) was reviewed. Following this literature review, we combined various factors to propose a practical methodology. We employed a multiple-criteria decision-making (MCDM) model to prioritize the factors affecting organ donation. Many MCDM calculation methods can be used to derive values for prioritization, thereby solving decision-making problems. The analytic hierarchy process (AHP), proposed by Stoeckle [20], was designed for supplier selection and involves compiling comparative evaluation criteria of supplier performance; the AHP has been used widely to solve complex real-world problems. The AHP typically considers the unidirectional relationships among the factors and structures in the problem as a hierarchy. By contrast, if the problem context is a network where goal, criteria (and, where applicable, subcriteria), and alternatives are considered, the analytic network process (ANP) considers such factors to be nodes of the network, with bidirectional relationships.

Therefore, this study employed the ANP as the basic framework and used scientific modeling to explore the factors affecting the decisions of families regarding donating organs of family members in an ICU. In the ANP framework, the relationships between and the weights of diverse factors were compared and ranked on the basis of importance. The findings can offer assistance to organ procurement programs, enabling greater success in organ procurement to be achieved. The purpose of this study was to identify the prominent psychological drivers of patients' families providing consent on behalf of ICU patients regarding organ donation; to this end, the following research questions were addressed:

1. What are the prevailing attitudes of the families of ICU patients in relation to organ donation?
2. What are the main factors affecting family acceptance of ICU patients' organ donation?
3. What is the priority level of each identified factor influencing organ donation consent?

## 2. Literature Review

Organ transplantation is a treatment method for end-stage organ failure whereby a patient's life is extended and quality of life is improved. Organ donation refers to the donation of body organs or tissues, which are surgically removed from a donor and transplanted to one or multiple recipients. In real-world settings, three types of donation systems are commonly used in the procurement of organs: (1) the opt-out (presumed consent), (2) opt-in, and (3) presumptive approaches. The findings of different countries after implementation of these systems imply that their effectiveness largely depends on how the systems address the factors affecting the willingness to donate, which may include educational, cultural, and social backgrounds [10]. Organ donation is a sensitive topic, particularly from a traditional Chinese cultural perspective and in relation to patients who are at the end stage of their lives. Despite studies not having reached a consensus on the factors influencing the decision to donate organs, several candidate factors have been proposed and can be categorized into demographic, physiological, psychological, spiritual, and external factors as follows.

### 2.1. Demographic Factors

Araujo and Siqueira [11] and Goz et al. [12] asserted that age does not affect attitude toward organ donation, but Cohen et al. [13] reported that age and attitude were significantly positively correlated. Furthermore, in one study, women were more positive about organ donation than men [14], whereas Siminoff, Gordon, Hewlett, and Arnold argued that men are more likely to donate organs because they bear greater responsibility than women from the perspective of traditional ideals [8]; Jung reported no differences in organ donation based on sex [15].

Numerous studies have suggested that educational attainment influences intention regarding organ donation [11, 16]. Pouraghaei et al. [16] also reported that individuals in full-time employment were more likely to have organ donation intention. Akgun et al. [17] observed that respondents with a medical background were more likely to intend to donate than those with a background in another profession. Finally, organ donation intention tends to be less prevalent in close-knit families because family members cannot bear to damage the remains of loved ones or refuse donation to avoid intrafamily conflict [11].

### 2.2. Physiological Factors

Siminoff et al. [18] reported that family-decided organ donation was more prevalent (65.1%) when the patient died of external trauma. Thus, a correlation may exist between cause of death and organ donation intention. In Asia, preserving the remains of the deceased, particularly their sensory organs, is a long-standing custom. In clinical settings, the family commonly agrees to donate any part of the deceased except the corneas in accordance with the rationale that the deceased will be unable to journey to the afterlife effectively if deprived of eyesight. However, Siminoff et al. [18] reported that the consent of the family was unaffected by the body part desired for donation.

### 2.3. Psychological Factors

If the deceased has not left a will or an advance directive, the family of the deceased is granted legal ownership of the deceased's remains. Therefore, the family's attitude is a major factor affecting the decision regarding organ donation. Numerous studies have confirmed that individuals with a positive attitude toward organ donation are more likely to have organ donation intention [7, 19, 20]. Nursing personnel in ICUs generally has a positive attitude toward organ donation, and patients' families who consult nurses on such matters may be influenced by their positive attitude.

### 2.4. Spiritual Factors

Hsieh et al. [21] listed a number of causes for patients' families refusing organ donation, including traditional customs, family concerns, value systems, cognitive differences, and organs being deemed medically unsuitable for transplantation; they identified custom as the primary cause of most people's traditional belief that the remains of the deceased must be left intact or fear of bringing greater suffering (e.g., mutilation) to their loved one after death. Davison and Jhangri [22] concurred that cultural beliefs have a considerable effect on organ donation intention. Holman et al. [23] further delineated the effects according to religious belief; Catholics (77%) and Orthodox Christians (73%) were more likely to have organ donation intention than Protestants (43%). Conversely, Goz et al. [12] reported that religious belief does not affect people's organ donation decision. In the Netherlands, Witkamp et al. [24] interviewed the families of critically ill patients and reported that those who had discussed death with the patient were more open to the idea of organ donation than those who had not. Simpkin et al. [25] and Wu [26] both noted that discussing death with family members gives individuals more insight into death, reduces their anxiety about death, and affects their intention regarding organ donation.

### 2.5. External Factors

Organ procurement typically involves medical professionals explaining the relevant details to a patient's family in a quiet place. Gortmaker et al. [27] observed that conducting such discussions in a nursing station offered a greater likelihood of success than in the corridor or the ward (56%, 52%, and 30%, respectively). Simpkin et al. [28] contended that, if possible, organ procurement dialogue with families should be conducted in a secluded place to improve the likelihood of success. Niles and Mattice [29] conducted a retrospective study and noted that although attempting organ procurement discussion before versus after the death of a patient did not exert a significant effect on the granting of consent, doing so immediately upon the death of a patient reduced family consent to 32%–37%. Instead, the ideal time for the organ procurement discussion was the point at which brain death was declared (65.4%).

## 3. Analytic Network Process

This study employed the ANP as its main framework to analyze the factors that influence the organ donation decisions of patients' families. To resolve problems involving uncertainty and multiple criteria, Saaty [30] developed the AHP to prioritize such criteria in decision-making. The AHP uses stratified and independent approaches to solve complex decision-making problems by identifying the weights of decision alternatives by using quantified calculation methods. However, decision-making problems are highly diverse and complex, and one limitation of the AHP is that the factors that can influence a decision must be independent. Therefore, in some cases, the AHP is not applicable. To address this deficiency, Saaty extended the AHP to develop a new decision-making framework: the ANP. The ANP has been described as a special case of the AHP [31]. The AHP considers the unidirectional relationships among the factors and structures in the problem as a hierarchy, whereas the ANP structures the problem context as a network in which the goals, criteria (and, where applicable, subcriteria), and alternatives are considered nodes of the network. Thus, unlike the AHP, the ANP allows for loops and feedback between nodes to represent interdependency among the factors. The ANP is based on the pairwise comparisons of the AHP whereby criteria are compared with each of the decision alternatives, necessitating an additional set of comparisons where alternatives are pairwise-compared against each criterion. The ANP allows interactions and feedback among decision criteria to be included through the introduction of evaluation scales into the decision model. The ANP can systematically solve problems involving multiple decision-making criteria by employing a nonlinear network structure based on the problem type [31]. Moreover, the ANP is commonly used to solve multiple-criteria decision problems that cannot be defined using a hierarchical structure, such as product planning, strategic decision-making, and other multidimensional analyses. In these cases, relations are found not only among criteria in the same hierarchy but also among criteria in different hierarchies. Therefore, the ANP was the more appropriate framework than the AHP, given our research goal, and it was adopted in this study accordingly.

The main purposes of developing a network structure were to confirm the problem, clearly describe and identify the decision criteria, define the factors involved with each criterion and subcriterion, identify the interrelations among the criteria, and graph the ANP model. The flow chart of the proposed approach is given in Figure 1. There are four major steps in the ANP, namely, (1) development of a network structure and creation of pairwise comparison matrices, (2) calculation of the relative weights of those matrices, (3) construction of a supermatrix, and (4) selection of the best solution [31]. In accordance with the recommendation of Saaty [31], the following steps should be followed to perform the ANP.

### 3.1. Developing Pairwise Comparison Matrices

Saaty [31] asserts that the relative importance of *n* factors (i.e., subcriteria) with respect to a specific element in the immediate upper level should be assessed through a pairwise comparison that utilizes a 9-point scaling system. Patients' families were the targeted respondents for the pairwise matrix comparisons. The pairwise comparison matrices were constructed, the relative importance and weights of the criteria were calculated, and pairwise comparisons of the criteria were made on the basis of a scale from 1 to 9, as detailed in Table 1. The comparisons included comparisons of criteria with factors and comparisons among factors, which included comparisons among factors of the same criterion and among factors of different criteria. The participants were invited to compare two criteria, or two factors—say A and B—in a certain situation. If they believed A was more important than B, they recorded a score of 5–9 on the scale. If they disagreed that A was more important, they recorded a score of 1–4.

### 3.2. Normalizing the Matrices and Obtaining Priority Vectors

The results of each pairwise comparison were arranged in a pairwise comparison matrix (**W**). Matrix **W** was normalized by dividing each element of the matrix by its column sum. To obtain a priority vector, the rows of **W** were averaged using the arithmetic mean.

### 3.3. Evaluation of Consistency

Similarly, after the participants had given answers for all items, the obtained data were used to create *n* × *n* comparison matrices. To prevent errors in the research results, the comparison matrices were strictly consistent before and after. Thus, evaluating the consistency of the scale results by using the consistency index (CI) and consistency ratio (CR) was essential. This was how the consistency of the potential decisions made could be assured. The decision-makers' decisions were consistent when the CR was under 0.1.

### 3.4. Developing the Weighted Supermatrix

After confirming the consistency by using the CI and CR, the eigenvector of each matrix was obtained and used as the weight of the given matrix. An unweighted supermatrix could be constructed using the weight of each matrix according to the interrelations of the factors. Then, the supermatrix was normalized to create the weighted supermatrix. This supermatrix could efficiently solve the problem of criterion dependence. It was composed of multiple submatrices. Each submatrix was composed of the interrelations among the relevant factors. By comparing it with the other matrices, the corresponding eigenvectors could be obtained as the weight of the submatrix. The convergent values of the limit supermatrix were the weights of the corresponding criteria, and these weights represented the relative importance of the criteria (constructs) and factors used to evaluate the alternatives for the research problem. The alternatives could then be prioritized on the basis of these weights.

## 4. Methods

In this study, a literature review was performed to identify factors affecting the organ donation attitude of families with a member in an ICU. In the first step, we adopted a cross-sectional questionnaire to examine the attitude of the respondents; then the findings were integrated with our clinical experience to produce study variables of the ANP questionnaire to investigate the patient's families with a positive attitude who are more likely to donate organs by the ANP framework questionnaire in the second step. Because the research framework was based on the ANP in this study, the Super Decision 2.6.0 (http://www.superdecisions.com/) and WEKA 3.8.0 open-source data mining (http://www.cs.waikato.ac.nz/ml/weka/) software packages were used to calculate the dependence and feedback between the constructs and factors, upon which the weights of factors were determined to establish a decision tree.

### 4.1. Samples

Participants were recruited from five types of ICU—the subacute respiratory, medical, neurosurgery, surgical, and cardiac ICUs—of a regional teaching hospital in Taiwan. Each participant, who was the main decision-maker in the respective patient's family, was required to indicate his/her attitude toward organ donation by using a Likert Scale. Then, quartile clustering was performed to select a most positive group to answer the ANP questionnaire with 4 constructs and 18 factors pertaining to organ donation. When estimated using *G*^*∗*^Power 3.1 with a significance level of 0.05, power of 0.80, and effect size of 0.15, the minimum sample size required was determined to be 150 participants [32]. In consideration of some questionnaires potentially not being returned, this study's sample size was determined as 180 participants.

The inclusion criteria were (1) being the main decision-maker in the family of a patient in an ICU and (2) being an adult aged ≥20 years. The exclusion criteria were (1) having received a diagnosis of a mental disorder and (2) being deaf or mute or having comprehension impairment. Discussing the prospect of participating in the study with ICU patients' family members was difficult when they were at the bedside of the patient, in a bad mood, or feeling rushed. Hence, observing the sentiment of patients' families first and then selecting an appropriate and comfortable time to ask for their participation in our study were essential. We spent nearly 1 year collecting all the study questionnaires. Fortunately, only eight individuals declined our request to participate before the desired 180 completed questionnaires were obtained.

### 4.2. Research Process

The research process of the present study comprised three phases. First of all, the topic was determined, and a thorough understanding of the relationship of the variables was gained on the basis of literature review and our clinical experience. In the second phase, after literature review was conducted, variables were identified and scales appropriate for assessing attitude toward organ donation were collected to establish the ANP questionnaire of this study. In the third phase, the organ donation attitude questionnaire and the ANP questionnaire were combined to perform an investigation on the factors affecting the organ donation decisions.

### 4.3. Research Instrument

The research instrument was self-developed on the basis of the results of literature review and our own clinical experience. It addressed three aspects, namely, demographic attributes, attitude toward organ donation, and factors affecting the organ donation decision of families with a member in an ICU. The demographic attributes recorded were age, gender, marital status, educational attainment, occupation, and religious belief as well as family relations and relationship with the patient. The organ donation attitude questionnaire was compiled by Yen [33]. It was employed to gauge the participants' attitudes toward organ donation. Specifically, the questionnaire consisted of eight items covering egoism, altruism, and constraints and exhibited a Cronbach's *α* of 0.84. A Likert Scale was used for scoring, with a high score denoting a positive attitude.

In the third phase of the research process, we developed a questionnaire inquiring into the factors affecting the organ donation decisions of families with a member in an ICU by applying the ANP method based on experience and the results of the literature review. The 1–9 scoring system proposed by Saaty [31] was adopted for pairwise comparisons. The initial draft of the questionnaire, which consisted of 18 factors associated with 4 constructs, was reviewed by six experts, who provided valuable feedback and rated the items by their relevance and appropriateness in relation to language and scoring. The content validity index of the items averaged 0.87, exceeding the benchmark of ≥0.8 [34]. The method also calculates a consistency ratio (CR) to verify the coherence of the judgments, which must be about 0.10 or less to be acceptable. Mathematical foundations of the AHP can be found in Saaty [31]. The questionnaire was then issued to participants for data collection.

### 4.4. Ethical Considerations

This study was approved by the institutional review board of E-Da hospital (approval no: AF08-008). Before answering the questionnaire, the participants were comprehensively informed of their rights and the purpose of the study and were also required to sign an informed consent form. To protect the rights of the ICU patients and their families, the questionnaire was anonymous, and identifiers such as patient identification codes were encoded with serial numbers such that individuals could not be identified.

## 5. Results

A cross-sectional research design was adopted to explore the factors affecting the organ donation decision of families with a member in an ICU. A total of 180 participants were included; among them, 68.9% were females, 66.1% were married, and 57.8% had an educational attainment of college or higher. Service industries were the most prevalent occupation, accounting for 36.1% of the participants. The participants were aged 21–87 years, with a mean age of 40.43 years. In terms of religious belief, most participants were either Taoist (69; 38.3%) or Buddhist (49; 27.2%). Regarding their relationships with the patient, 20 (11.1%), 18 (10%), 26 (14.4%), and 75 (41.7%) participants were the patient's parent, sibling, partner, and child, respectively. Most of the participants (96.7%) reported their family relations as being close. Only 15 (8.3%) participants reported that the ICU patient from their family had signed an organ donor card. Most of the participants (117; 65%) were positive about organ donation, but only 39 (21.7%) had discussed organ donation with other family members. A total of 115 (63.9%) participants asserted that they would support their family members' decision to donate their organs at their time of death.

In the organ donation attitude questionnaire, the participants gave scores of 31.67 ± 5.34 out of 40 (a higher score indicated a more positive attitude). Detailed information is presented in Table 2.

The results of bivariate analysis indicated that age and attitude toward organ donation were significantly negatively correlated (*r* = −0.221 and *p* = 0.003). Other parameters that significantly correlated with organ donation attitude were gender, marital status, educational attainment, family relations, and responses to the following questionnaire items: “*Have you signed an organ donor card?*,” “*Do you agree that organ donation is a personal decision?*,” “*Have you discussed organ donation with the patient?*,” and “*Do you agree with the patient's organ donation intention and attitude toward organ donation?*” The results of one-way analysis of variance indicated that occupation (*F* = 1.556 and *p* = .152), religious belief (*F* = 1.091 and *p* = .362), and the relationship with the patient (*F* = 1.571 and *p* = .171) were not significantly correlated with attitude toward organ donation or organ donation intention.

Clustering was performed with the scores obtained using the organ donation attitude questionnaire. Quartile clustering was applied to the attitude scores, and the cluster with the highest score (*n* = 50) was selected for an ANP-based analysis to determine the main factors affecting the organ donation decision of the participants who held a positive attitude toward organ donation. Pairwise comparison was conducted on the factors in the four constructs to establish factor weights on the basis of the internal dependence they exhibited.  Table 3 presents the priority values of the factors associated with attitude toward organ donation; the factors were ranked by importance. The table thus reveals the constructs and factors that play a major role when a patient's family must make a decision regarding organ donation.

A limit supermatrix, which was obtained from the computation results of Super Decisions, was used to determine the order of priority of the constructs and factors (Figure 2). All the criteria and subcriteria and the details are given a code letter. There, codes given in tables 4 and 5 will be used in the supermatrix. The weights in Table 3 were sorted, revealing the psychological construct (0.475751) as the most influential, followed by the external factors (0.203193) and spiritual (0.197258), and physiological (0.123799) constructs. For the psychological construct, the factor receiving the highest priority was attitude toward organ donation (0.31589). For the external factor's construct, the key factor was the physician's care experience (0.008866); for the spiritual construct, the key factor was religious belief (0.192601); for the physiological construct, the main factor was organ selection (0.31903). In summary, attitude toward organ donation (part of the psychological construct) was the most critical factor, whereas organ selection (a physiological construct) was the least critical factor.

The results of the clusters with the highest score were computed in WEKA software version 3.8.3 to investigate the classification and establishment of the decision tree by the C.4.5 [35], cart [36], and random tree [37] classifiers. The experimental results indicated that the random tree algorithm was the most suitable classifier. Therefore, random tree was used for the development of the decision tree, which could aid clinical procurement transplant coordinators in deciding when to discuss organ donation with ICU patients' families.  Figure 3 illustrates the resultant decision tree, from which a set of if-then classification criteria, namely, a decision factor priority list of agreeing with organ donation, is generated as follows:

- If psychological factors are satisfied = Y, physiological factors are satisfied = Y, and external factors are satisfied = Y, then organ donation = agree.
- If psychological factors are satisfied = Y, physiological factors are satisfied = N, and spiritual factors are satisfied = Y, then organ donation = agree.
- If psychological factors are satisfied = N and external factors are satisfied = Y, then organ donation = agree.

## 6. Discussion and Conclusion

This study investigated factors affecting the attitude of families of a member in an ICU regarding organ donation. The results indicated that organ donation attitude was correlated with age. Educational attainment, whether the patient had signed an organ donor card, and attitude toward organ donation were significantly correlated with families' consent to organ donation.

This study primarily applied the ANP to identify the factors affecting the decisions of ICU patients' families regarding organ donation. This study exhibited some limitations in relation to the selection of methodology and data collection. First of all, the ANP-based questionnaire used in this study was markedly different from conventional questionnaires and required step-by-step explanation, which considerably prolonged the time required to obtain responses. Consequently, the answers may not have accurately reflected the participants' consideration in decision-making, thus compromising the results. Furthermore, because the study was cross-sectional and predictive, the results may be inapplicable to other organ donation settings. Another concern is that the participants were recruited at a single hospital, rendering the results potentially unsuitable for extrapolation to other populations. Moreover, the most obvious limitation of the research is the subjectivity due to the use of surveys. All the opinions about organ donation and relative importance are obtained from the questionnaire, and the research results are greatly dependent on the relative knowledge and experience of the patients' families. Although a scientific approach was used, only using pairwise comparison of factors compiled in advance could not thoroughly reflect the feelings of family members. Nevertheless, we contend that the key features of this study were the proposed MCDM model and preliminary understanding of the attitude of ICU patients' families. Future research should employ a qualitative method to explore the views of patients' families on the meaning and value of organ donation when their relative's organs are removed for transplantation. Through a more in-depth analysis, additional factors that directly and indirectly influence patients' families in their organ donation decision-making should be identified. In clinical settings, we advise that medical institutions should host workshops related to organ donation and transplantation more often. Such workshops would enable personnel from various backgrounds to share their experiences, facilitate discussion, and enable members of an organ procurement team to better understand each other's roles, optimize use of team resources, build a consensus, increase the likelihood of successful organ donation, and save more patients requiring organ transplant.

## Figures and Tables

**Figure 1:** Process flowchart for organ donation decision-making with ANP methodology.

**Figure 2:** Network structure of ANP.

**Figure 3:** Decision tree for organ donation of ICU patient's family.

**Table 1:** Pairwise comparison for AHP or ANP preferences.

Importance	Definition	Explanation
1	Equal importance	Two activities contribute equally to the objective.
2	Weak or slight	

3	Moderate importance	Experience and judgment slightly favor one activity over the other.
4	Moderate plus	

5	Strong importance	Experience and judgment strongly favor one activity over the other.
6	Strong plus	

7	Very strong or demonstrated importance	One activity is very strongly favoured over the other; its dominance is demonstrated in practice.
8	Very, very strong	

9	Extreme importance	The evidence favoring one activity over the other is of the highest possible order of affirmation.

**Table 2:** Descriptive statistics of attitude about organ donation.

Positively/negatively	Items	*μ* ± *σ*
Positively worded items	“*Organ donation is a good thing and the right thing.*	4.30 ± .776
	*Donating the organs of a loved one makes me feel they are still alive; it is a continuation of their life.*	4.14 ± .891
	*Organ donation helps others by saving their lives.*	4.39 ± .728
	*Organ donation is an expression of altruistic love.*	4.21 ± .784

Negatively worded items	*I do not want to donate the organs of my loved one because I am worried about the opinions of family and friends.*	3.47 ± 1.043
	*I do not want to donate the organs of my loved one because I'm worried that the hospital would not do their best in saving my loved one.*	3.66 ± 1.099
	*Donating organs means the remains of my loved one will be incomplete; that is why I reject it.*	3.74 ± 1.015
	*Our bodies—to every hair and bit of skin—are received by us from our parents, and we must not presume to injure or wound them; that is why organ donation is unacceptable.*	3.74 ± 1.015

**Table 3:** Weights of constructs and factors of decision-making for organ donation.

Constructs	Factors	Factor's weight	Priority of factor	Construct's weight	Rank of dimension
Spiritual	Faith	0.192601	V	0.197258	3
	If mention dead issue with family	0.038521			

Physiological	Organ selection	0.31903	V	0.123799	4
	Cause of death	0.05139			

External	Transplant coordinator background	0.003948		0.203193	2
	Organ procurement timing	0.003190			
	Nursing care experience	0.005554			
	Physician care experience	0.008866	V		
	Hospital ranking	0.001857			
	Hospital reputation	0.002569			
	Privacy environment	0.001858			

Psychological	Positive attitude	0.31589	V	0.475751	1
	Negative attitude	0.31589			

**Table 4:** Unweighted supermatrix in the ANP model.

	Constructs	Spiritual		Physiological			External						Psychological	
Constructs	Factors	1	2	3	4	5	6	7	8	9	10	11	12	13
Spiritual	Faith (1)	0	1	0.75	0.8	0.8	0.75	0.8	0.833	0.8	0.833	0.833	0.857	0.8
	If mention dead issue with family (2)	1	0	0.25	0.2	0.2	0.25	0.2	0.167	0.2	0.167	0.167	0.143	0.2

Physiological	Organ selection (3)	0.197	0.197	0.875	0.197	0.125	0.197	0.197	0.197	0.197	0.197	0.197	0.197	0.197
	Cause of death (4)	0.051	0.051	0.125	0.051	0	0.051	0.051	0.051	0.051	0.051	0.051	0.051	0.051

External	Transplant coordinator background (5)	0.1	0.167	0.333	0.167	0.017	0	0.128	0.158	0.08	0.083	0.148	0.09	0.09
	Organ procurement timing (6)	0.752	0.752	0	0.752	0.875	0.752	0.752	0.752	0.752	0.752	0.752	0.752	0.752
	Nursing care experience (7)	0.108	0.167	0	0.167	0.107	0.138	0	0.179	0.146	0.229	0.269	0.148	0.149
	Physician care Experience (8)	0.136	0.167	0	0.167	0.519	0.209	0.222	0	0.22	0.145	0.413	0.209	0.21
	Hospital ranking (9)	0.186	0.167	0.333	0.167	0.035	0.055	0.054	0.147	0	0.054	0.067	0.045	0.063
	Hospital reputation (10)	0.216	0.167	0	0.167	0.071	0.085	0.08	0.103	0.051	0	0.103	0.062	0.042
	Privacy environment (11)	0.254	0.167	0.333	0.167	0.252	0.513	0.517	0.412	0.503	0.489	0	0.447	0.446

Psychological	Positive attitude (12)	0.875	0.833	1	1	0.5	0.5	0.5	0.5	0.5	0.5	0.5	0	1
	Negative attitude (13)	0.125	0.167	0	0	0.5	0.5	0.5	0.5	0.5	0.5	0.5	1	0

**Table 5:** Weighted supermatrix in the ANP model.

	Constructs	Spiritual		Physiological			External						Psychological	
Constructs	Factors	1	2	3	4	5	6	7	8	9	10	11	12	13
Spiritual	Faith (1)	0	0.04	0.12	0.13	0.13	0.36	0.38	0.39	0.38	0.39	0.39	0.17	0.16
	If mention dead issue with family (2)	0.04	0	0.04	0.03	0.03	0.12	0.09	0.08	0.09	0.08	0.08	0.03	0.04

Physiological	Organ selection (3)	0.02	0.02	0.12	0.03	0.02	0.01	0.01	0.01	0.01	0.01	0.01	0.01	0.01
	Cause of death (4)	0	0	0.02	0.01	0	0	0	0	0	0	0	0	0

External	Transplant coordinator background (5)	0.05	0.08	0.13	0.07	0.01	0	0.01	0.02	0.01	0.01	0.02	0.01	0.01
	Organ procurement timing (6)	0.07	0.07	0	0.1	0.12	0.04	0.04	0.04	0.04	0.04	0.04	0.04	0.04
	Nursing care experience (7)	0.05	0.08	0	0.07	0.04	0.02	0	0.02	0.02	0.03	0.03	0.01	0.01
	Physician care Experience (8)	0.07	0.08	0	0.07	0.21	0.02	0.02	0	0.02	0.02	0.05	0.02	0.02
	Hospital ranking (9)	0.09	0.08	0.13	0.07	0.01	0.01	0.01	0.02	0	0.01	0.01	0	0.01
	Hospital reputation (10)	0.11	0.08	0	0.07	0.03	0.01	0.01	0.01	0.01	0	0.01	0.01	0
	Privacy environment (11)	0.13	0.08	0.13	0.07	0.1	0.06	0.06	0.05	0.06	0.05	0	0.04	0.04

Psychological	Positive attitude (12)	0.19	0.18	0.11	0.11	0.06	0.11	0.11	0.11	0.11	0.11	0.11	0	0.43
	Negative attitude (13)	0.03	0.04	0	0	0.06	0.11	0.11	0.11	0.11	0.11	0.11	0.43	0

## Data Availability

The data used to support the finding of this study are included within the article.
